The article "Protective effect of erythropoietin against myocardial injury in rats with sepsis and its underlying mechanisms" was retracted in 2025. Reasons: duplicated images; overlap with earlier publications; concerns about the images; concerns about the citations.

# Protective effect of erythropoietin against myocardial injury in rats with sepsis and its underlying mechanisms

**DOI:** 10.3892/mmr.2015.3155

**Published:** 2015-01-08

**Authors:** XINLIANG ZHANG, SHIMIN DONG, YANJUN QIN, XIAOHUA BIAN

**Affiliations:** 1 Department of Emergency, The Third Hospital of Hebei Medical University, Shijiazhuang, Hebei 050051, P.R. China; 2 Department of Critical Care Medicine, The Third Hospital of Hebei Medical University, Shijiazhuang, Hebei 050051, P.R. China

**Keywords:** sepsis, myocardial injury, erythropoietin, apoptosis

## Abstract

The aim of this study was to investigate the protective effect of erythropoietin (EPO) against acute myocardial injury and its underlying mechanisms. Mice (n=146) were randomly divided in a double-blind manner into four groups, sham, Rocephin, EPO and sepsis, and mortality was observed on the seventh day after cecal ligation and puncture. In addition, a total of 252 rats were randomly divided into three groups, sham, EPO and sepsis, and indicators of cardiac function, inflammatory mediators and serum creatine kinase levels were assessed. Mitochondrial membrane potential, cell apoptosis and nuclear factor κ-light-chain-enhancer of activated B cells (NF-κB) p65 expression levels were detected using flow cytometry. Following intervention with EPO, the mortality rate in mice with sepsis was significantly reduced and the cardiac function of septic rats was significantly improved. In addition, the levels of inflammatory mediators, serum creatine kinase and apoptosis and the myocardial mitochondrial membrane potential and expression of NF-κB p65 in cardiac tissue were all improved following EPO treatment, and the differences between the results for the sepsis and EPO groups were statistically significant (P<0.05). These findings suggest that EPO reduces the myocardial inflammatory response in septic rats, attenuates the reduction in mitochondrial membrane potential and inhibits myocardial cell apoptosis by reducing NF-κB p65 expression, and therefore exerts a protective effect in the myocardium.

## Introduction

Sepsis is a systemic inflammatory response syndrome (1) caused by any pathogenic factor and is an important cause of multiple organ dysfunction syndrome (MODS). During the progression of sepsis, inflammatory mediators and cytokines are released following exposure to harmful stimuli, resulting in host autoimmunity injury (2). The mortality rate of severe sepsis and septic shock is ≤50%, and the incidence rate is increasing progressively every year (3,4). The incidence of myocardial depression in severe sepsis is ≤80% and the incidence of myocardial injury is ≤40%, which severely affects the prognosis of patients (5). The administration of positive inotropic drugs can improve the ejection fraction of the heart; however, myocardial oxygen consumption is likely to also increase, and therefore the net benefit is unknown. At present, there is no effective method for improving myocardial depression; thus, a novel therapeutic approach is required.

The article "Protective effect of erythropoietin against myocardial injury in rats with sepsis and its underlying mechanisms" was retracted in 2025. Reasons: duplicated images; overlap with earlier publications; concerns about the images; concerns about the citations.

In myocardial injury during sepsis there is a decline in cardiac function. This decline in cardiac function is an important mechanism for refractory hypotension, which seriously affects the prognosis of sepsis. For the treatment of sepsis, the timely administration of antibiotics can effectively kill pathogens to reduce the rate of mortality (3). In the present study the antibiotic Rocephin was used as a positive control to observe the mortality of Kunming mice with sepsis.

Cytokines can act in either a pro- or anti-inflammatory manner. The group of proinflammatory cytokines has been shown to include tumor necrosis factor α (TNF-α), interleukin 6 (IL-6) and IL-8, while the anti-inflammatory cytokines, which inhibit the inflammatory response, include IL-10. The interactions and dynamic balance between pro- and anti-inflammatory cytokines play an important role in maintaining the stable internal environment of the body; in certain cases an imbalance can result in an increase in the inflammatory response and organ dysfunction, leading to the occurrence of MODS (6). When sepsis occurs, nuclear factor κ-light-chain-enhancer of activated B cells (NF-κB) is activated in the inflammatory cells, leading to a heightened, uncontrollable inflammatory reaction. The activated inflammatory cells release large numbers of pro- and anti-inflammatory cytokines, resulting in an imbalance in cytokine levels, and therefore causing organ dysfunction and inflammatory injury to the tissue (7).

Programmed cell death, known as apoptosis, is a type of cell death that occurs during the processes of body morphogenesis, tissue remodeling and immune response retrogression, and is the pathological process underlying the development of sepsis (8). Tramontano *et al* (9) and Maiese *et al* (10) reported that, when erythropoietin (EPO) binds to its receptor on the cell surface, the receptor becomes activated. EPO, a glycoprotein, which stimulates the bone marrow hematopoiesis, is a member of the type I cytokine family with a molecular weight of 30.4 Kda. EPO is mainly synthesized and secreted by renal tubular juxtaglomerular cells at the junction of the renal cortex and medulla (4–6).

EPO promotes erythrocytopoiesis. The function of hematogenesis is to promote hematopoietic erythroid progenitor cells to differentiate into mature red blood cells, thereby increasing the number of red blood cells in the circulation and the concentration of hemoglobin (11). In addition to findings regarding the role of EPO in the circulatory system, it has been observed that EPO receptors are widely distributed in non-hematopoietic tissues, including broad expression in the cardiovascular system of EPO and EPO-R (9). These findings suggest that EPO has a variety of non-hematopoietic biological effects in addition to protective effects in the cardiovascular system, including as a hematopoietic growth factor (12). EPO protects endothelial cells, and inhibits apoptosis of cardiomyocytes and immune cells, which has a protective effect on cells in animal and human models of the ischemic injury (13). The present study aimed to investigate apoptosis in sepsis and the role of EPO in the sepsis anti-apoptotic process.

The article "Protective effect of erythropoietin against myocardial injury in rats with sepsis and its underlying mechanisms" was retracted in 2025. Reasons: duplicated images; overlap with earlier publications; concerns about the images; concerns about the citations.

This results in the activation of protein kinase B and signal transduction through Janus kinase 2 and phosphatidylinositol 3,2 kinase, leading to alterations in the activity of downstream signaling molecules. Consequently, the stability of the mitochondrial membrane potential can be maintained, which results in a decrease in the release of cytochrome *c* and the inhibition of caspase-3 activation. Therefore, EPO has a biological role in the inhibition of apoptosis. In eukaryotes adenosine triphosphate is generated by oxidative phosphorylation in the mitochondria, and maintaining the mitochondrial transmembrane potential is essential for mitochondrial function. When the potential difference between the inside and outside of the mitochondrial membrane is reduced, i.e. the mitochondrial membrane potential is decreased, a series of biochemical changes occurs inside and outside of the mitochondrial membrane, including changes in mitochondrial membrane permeability, the extensive release of cytochrome *c* and the activation of the B-cell lymphoma 2 family and caspases. This activates the apoptosis cascade reaction leading to apoptosis (14,15). When the decrease in mitochondrial membrane potential is effectively inhibited, the incidence of cell apoptosis is reduced. Therefore, a reduction in mitochondrial transmembrane potential is considered to be one of the irreversible events that occur during apoptosis and in early apoptotic cells (15–17).

Cytokines are not stored in the cells, but are generated by gene transcription, translation and protein modification. The transcriptional process is an important mechanism in the regulation of cytokine production during inflammatory reactions. Nuclear transcription factors are one of the key factors in the generation of inflammatory mediators, in particular NF-κB. The gene expression of a number of cytokines, as well as adhesion and chemoattractant molecules, is regulated by NF-κB, which has an important role in the pathogenesis of the sepsis (18,19).

The article "Protective effect of erythropoietin against myocardial injury in rats with sepsis and its underlying mechanisms" was retracted in 2025. Reasons: duplicated images; overlap with earlier publications; concerns about the images; concerns about the citations.

Sepsis causes myocardial depression and injury, and, at present, there is no effective therapeutic treatment against myocardial depression. Therefore, in the present study, a rat model of sepsis with myocardial injury was established using cecal ligation and puncture (CLP), and the protective effect of EPO was investigated. The effects of EPO were studied from a physiological, pathological and molecular perspective, and indicators of cardiac function, the inflammatory response, serum creatine kinase (CK), myocardial histopathology and cardiomyocyte apoptosis were detected to determine whether EPO exerted a protective effect on the heart and other major organs (liver, kidney and lung) in sepsis. The molecular mechanism of EPO was also investigated to provide a theoretical basis for clinical therapeutic applications.

## Materials and methods

### Animals

A total of 146 male, clean-grade Kunming mice (6–8 weeks old, weighing ~20 g) and a total of 252 healthy male, clean-grade Sprague Dawley (SD) rats (weighing between 210 and 250 g) were used in the study. All the animals were provided by the Experimental Animal Center of Hebei Medical University (Shijiazhuang, China), were raised according to the requirements of clean-grade mice/rats and had free access to water. This study was performed in strict accordance with the Guide for the Care and Use of Laboratory Animals of the National Institutes of Health. The animal use protocol was reviewed and approved by the Institutional Animal Care and Use Committee of the Third Hospital of Hebei Medical University.

### Grouping of animal models

The grouping of animal models was divided into two parts: i) Grouping of healthy Kunming mice, which were used for the assessment of mortality rates following CLP surgery and ii) grouping of healthy SD rats, which were used for the observation of pathophysiological indicators following CLP surgery.

For the first part of the study, 146 Kunming mice were randomly divided in a double-blind manner into four groups: Sham (Sham, n=35), Rocephin (Roc, n=35), EPO intervention (EPO, n=35) and sepsis (CLP, n=35). A total of six mice succumbed to mortality and were, therefore, not included. For the observation of pathophysiological indicators, 252 healthy SD rats were randomly divided in a double-blind manner into three groups: Sepsis (CLP, n=8), EPO intervention (EPO, n=8) and sham (Sham, n=8). Of the 252 rats, 12 succumbed to mortality due to factors, including anaesthesia and temperature.

The article "Protective effect of erythropoietin against myocardial injury in rats with sepsis and its underlying mechanisms" was retracted in 2025. Reasons: duplicated images; overlap with earlier publications; concerns about the images; concerns about the citations.

### Establishment of the sepsis animal model

The animals were allowed to acclimate for one week subsequent to purchase and were fasted overnight before the start of the experiment, but with free access to water (n=8 per the Sham, EPO and CLP groups). The sepsis animal model was created using line CLP in accordance with a previously reported method (20).

Following the establishment of the sepsis model, EPO at a dose of 1,000 IU/kg was immediately and intraperitoneally injected into the animals in the EPO group and Rocephin at a dose of 1 mg/20 g was immediately intraperitoneally injected into the mice in the Roc group. In the Sham group, the abdominal cavity of the animals was opened and the abdominal incision was sutured once the cecum had been located; however, the cecum was not punctured.

### Cardiac hemodynamics

Following the CLP procedure, SD rat models from each group were taken at 0, 3, 6, 12 and 24 h. A catheter connected to a pressure transducer was inserted into the left ventricle of the heart via the common carotid artery. The pressure curve of the left ventricle was recorded, and the left ventricular systolic pressure (LVSP), the maximum rate of left ventricular pressure rise (+dP/dt_max_) and the maximum rate of left ventricular pressure decline (−dP/dt_max_) were calculated using the physiological recorder associated with Chart 4.0 software (eDAQ Pty Ltd., Denistone East, Australia).

### Preparation and storage of rat serum

Following the CLP procedure, SD rat models from each group were taken at 0, 3, 6, 12 and 24 h. Blood (5 ml) was obtained from the inferior vena cava for the detection of cardiac troponin I (cTnI), C-reactive protein (CRP), TNF-α, IL-6, IL-10, CK, aspartate aminotransferase (AST), and lactate dehydrogenase (LDH) using ELISA, in accordance with the manufacturer’s instructions.

### Preparation of single cell suspensions

SD rat models from each group were taken 24 h after the CLP procedure, and the fresh tissues (heart, liver, kidney and lung) were used to prepare single cell suspensions. The preparation of single cell suspensions was performed, as follows. Fresh tissues were placed onto a 120 mesh stainless steel net (The Fourth Hebei Medical University Hospital, Hebei, China) above a petri dish. The tissues were cut using ophthalmic scissors and gently rubbed with the scissors whilst rinsing with normal saline. The suspensions in the petri dish were filtered with a 300 mesh copper mesh filter (The Fourth Hebei Medical University Hospital) to remove cell clumps. The cell suspension was collected and precipitated by centrifugation at 829 × g for 2 min. The precipitate (single cell suspension) was collected, the supernatant was removed and the concentration was adjusted to 1×10^6^cells/ml.

The article "Protective effect of erythropoietin against myocardial injury in rats with sepsis and its underlying mechanisms" was retracted in 2025. Reasons: duplicated images; overlap with earlier publications; concerns about the images; concerns about the citations.

### Detection of apoptosis

Apoptosis was detected as previously described (21). A total of 100 μl cell suspension was taken and placed into 5-ml streaming tubes, prior to 5 μl Annexin V/fluorescein isothiocyanate and 10 μl propidium iodide (20 μg/ml) being added. The reaction was performed for 15 min in the dark at room temperature. A total of 500 μl buffer solution was subsequently added into the reaction tubes, and apoptosis was analyzed using flow cytometry (Epics of America XL II Flow Cytometry instrument; Beckman Coulter, Brea, CA, USA).

### Detection of mitochondrial membrane potential

A total of 100 μl rhodamine 123 was added to 0.1 ml single cell suspension with a concentration of 1×10^6^ cells/ml, and the cells were incubated for 30 min at room temperature in the dark. The cells were then washed with10 ml phosphate-buffered saline (PBS). The supernatant was subsequently removed and analyzed using flow cytometry (Epics of America XL II Flow Cytometry instrument).

### Detection of NF-κB p65

A total of 100 μl rabbit anti-rat NF-κB p65 primary antibody was added to 0.1 ml single cell suspension with a concentration of 1×10^6^ cells/ml, and the cells were incubated for 30 min at room temperature in the dark. The cells were then washed with 10 ml PBS and the supernatant was removed. A total of 100 μl secondary antibody working solution of goat anti-rabbit immunoglobulin G conjugated with horseradish peroxidase was added, and the cells were incubated for 30 min at room temperature in the dark. A total of 10 ml PBS was then added to the cells, prior to centrifugation. The supernatant was subsequently discarded to remove any unbound fluorescent secondary antibody, and 0.1 ml PBS filtered with 500-mesh copper mesh was added prior to detection using a flow cytometer. Background and negative controls for the primary and secondary antibodies were established when determining protein immunofluorescence markers. The samples were analyzed using flow cytometry (Epics of America XL II Flow Cytometry instrument).

### Production of light microscopy sections of rat tissues

Tissue sections were prepared using the conventional wax block method and stained with hematoxylin and eosin, prior to being observed and photographed under a light microscope.

### Statistical analysis

The data were analyzed using the SPSS 13.0 statistical software package (SPSS, Inc., Chicago, IL, USA) and all data are presented as the mean ± standard deviation. The inter-group differences were tested using the bilateral t-test for independent samples. P<0.05 was considered to indicate a statistically significant difference.

The article "Protective effect of erythropoietin against myocardial injury in rats with sepsis and its underlying mechanisms" was retracted in 2025. Reasons: duplicated images; overlap with earlier publications; concerns about the images; concerns about the citations.

## Results

### Mortality rates of mice seven days after CLP

Three hours after surgery, the sham-operated mice returned to a normal state. The rates of mortality in the mice in the Roc and EPO groups at 24 and 48 h were significantly reduced compared with those in the CLP group (P<0.01) (Table I and Fig. 1).

### Cardiac hemodynamic indicators

The LVSP, +dP/dt_max_ and −dP/dt_max_ values in the SD rats with sepsis were significantly decreased compared with those in the sham-operated rats (P<0.01). Rats in the CLP group exhibited decreases in the LVSP, +dP/dt_max_ and −dP/dt_max_ after 3 h, with the lowest values observed after 6 h. The values obtained in the CLP group were significantly lower than those obtained in the Sham group (P<0.01). The LVSP +dP/dt_max_ and −dP/dt_max_ values of the rats in the EPO group demonstrated partial restoration and were significantly higher compared with the values of the rats in the CLP group at 3, 6, 12 and 24 h (P<0.01) (Table II and Fig. 2).

### Comparison of inflammatory indicators

As shown in Table III, 6 h after the CLP, the CRP levels of the rats in the CLP and EPO groups peaked and were significantly increased compared with those of the rats in the Sham group (P<0.01). The CRP levels of the rats in the EPO and the CLP groups then progressively decreased; the difference between these two groups remained significant 12 h after the surgery (P<0.01).

Three hours after the CLP, the levels of TNF-α and IL-6 in the rats in the CLP and EPO groups peaked and were significantly increased compared with those in the rats in the Sham group (P<0.01). The levels of TNF-α and IL-6 in the rats in the CLP and EPO groups then progressively decreased and reached the lowest value 24 h after surgery; the difference between the two groups was significant (P<0.01).

Six hours after the CLP, the levels of IL-10 in the rats in the CLP and EPO groups peaked and were significantly increased compared with those in the rats in the Sham group (P<0.01). The levels of IL-10 in the CLP and EPO groups then showed a downward trend (Table III and Fig. 3).

### Comparison of indicators of myocardial enzymes

As shown in Table IV, the levels of cTnI in the SD rats in the CLP and EPO groups following the CLP were significantly higher than those in the rats in the Sham group, and were highest 12 h after the surgery (P<0.01). After 24 h the levels of cTnI decreased in the CLP and EPO groups; however, the levels in the EPO group were significantly lower than those in the CLP group (P<0.05).

Levels of CK increased 3 h after the CLP and then decreased at 6 h, prior to increasing again at 12 h and showing a continued increasing trend. Twelve hours after the CLP, the CK levels in the SD rats in the CLP and EPO groups were significantly higher than those observed in the Sham group (P<0.05).

The article "Protective effect of erythropoietin against myocardial injury in rats with sepsis and its underlying mechanisms" was retracted in 2025. Reasons: duplicated images; overlap with earlier publications; concerns about the images; concerns about the citations.

Following the CLP, the levels of AST and LDH in the SD rats increased progressively. Twelve hours after the CLP, statistically significant differences were observed in the levels of AST and LDH between the rats in the EPO group and those in the Sham group (P<0.01), and the serum AST and LDH levels were significantly lower in the rats in the EPO group than those in the rats in the CLP group (P<0.01) (Table IV and Fig. 4).

### Apoptosis

The results showed that 24 h subsequent to the CLP, the early and late apoptosis rates of the major organs (heart, liver, kidney and lung) of the CLP and EPO groups were significantly increased compared with those in the Sham group (P<0.01). The early apoptosis rate of the EPO group, however, was significantly lower than that of the CLP group (P<0.01) (Fig. 5A–D).

### Mitochondrial membrane potential

Twenty-four hours after the CLP, significant differences were observed in the mitochondrial membrane potential of the major organs (heart, liver, kidneys and lungs) between the CLP/EPO groups and the Sham group (P<0.01). When the CLP group was compared with the EPO group, the mitochondrial membrane potential of the major organs was shown to be significantly reduced (P<0.01). In the results from the flow cytometric analysis, the fluorescence peaks of the rat organ cells from the CLP and EPO groups were significantly shifted to the left when compared with those from the Sham group, i.e. the number of cells with low fluorescence intensity increased. This indicated that the mitochondrial membrane potential was significantly reduced (P<0.01).

Following treatment with EPO the fluorescence peaks of the rat cells from the EPO group were significantly shifted to the right compared with those from the CLP group, i.e. the number of cells with strong fluorescence intensity increased. This demonstrated that the reduction in mitochondrial membrane potential was significantly attenuated in the EPO group (P<0.01) (Fig. 6A–D).

### Expression of NF-κB p65

Twenty-four hours after the CLP, a significant difference was observed in the NF-κB p65 expression in the major organs (heart, liver, kidney and lungs) in the CLP and EPO groups compared with that in the Sham group (P<0.01). Comparing the EPO group with the CLP group, the expression of NF-κB p65 was significantly reduced (P<0.01) (Fig. 7A–D).

### Histopathology

Pathological sections of the rat hearts 24 h after the CLP are shown in Fig. 8A. In the Sham group, clear myocardial structure, well-arranged myocardial fibers, clear transverse striation and normal structure were observed. In the EPO group, however, the myocardial fibers had a wave-like arrangement with infiltration of inflammatory cells. In the CLP group, notable myocardial cell edema, as well as small, focal myocardial hemorrhage and focal myocardial necrosis were observed, with infiltration of a large number of inflammatory cells.

The article "Protective effect of erythropoietin against myocardial injury in rats with sepsis and its underlying mechanisms" was retracted in 2025. Reasons: duplicated images; overlap with earlier publications; concerns about the images; concerns about the citations.

Pathological sections of the rat livers 24 h after the CLP are shown in Fig. 8B. The Sham group exhibited complete hepatic lobule structure, normal liver cell morphology and no inflammatory cell infiltration. In the EPO group, the liver cell arrangement was slightly disordered, but the lobular structure remained intact. There was visible infiltration of inflammatory cells; however, the infiltration of inflammatory cells was milder than that observed in the CLP group. In the CLP group, the liver cells were swollen and disordered and there was visible infiltration of inflammatory cells.

Pathological sections of the rat kidneys 24 h after the CLP are shown in Fig. 8C. In the Sham group, normal tubular and interstitial morphology were observed, with no infiltration of inflammatory cells. In the EPO group, vacuolar degeneration was observed in the renal tubular epithelial cells, along with a small number of detached epithelial cells, but no significant edema in the renal interstitium. There was also visible infiltration of inflammatory cells in the renal interstitium, however, the infiltration was milder than that observed in the CLP group. In the CLP group, the kidneys had diffuse changes, with swelling and necrosis of the epithelial cells and caducous epithelial cells visible in small tubules. Glomerular capillary congestion was also observed and diffuse infiltration of a large number of inflammatory cells was detected in the renal interstitium, the extent of which was greater compared with the EPO group.

Pathological sections of the rat lungs 24 h after the CLP are shown in Fig. 8D. In the Sham group, the lungs were pink, with a smooth surface. The tissue exhibited normal swelling with no congestion or edema. Under the light microscope, normal alveolar structure with uniform alveolar septa (thin-walled and smooth) was observed, with no notable infiltration of inflammatory cells. In the EPO group, however, thickenings of the alveolar septa were observed, as well as the infiltration of inflammatory cells into the pulmonary interstitium and a small amount of oozing and bleeding in part of the alveolar space. However, the infiltration of inflammatory cells was less severe than that observed in the CLP group. In the CLP group, notable hyperemia and edema were observed in the lung tissue. The lungs were dark red on the surface, with light red liquid oozing on the incision surface and substantial alterations in the lung tissue. Under the light microscope, disordered alveolar structures, pulmonary capillary expansion and hyperemia were observed, as well as thickenings of the alveolar septa and visible oozing and bleeding in the alveolar space. In addition, significant inflammatory cell infiltration into the lung interstitium was apparent.

The article "Protective effect of erythropoietin against myocardial injury in rats with sepsis and its underlying mechanisms" was retracted in 2025. Reasons: duplicated images; overlap with earlier publications; concerns about the images; concerns about the citations.

## Discussion

In the first part of the present study, mice treated with Rocephin (Roc group) were used as a positive control group. The results showed that treatment with EPO significantly reduced the mortality of septic Kunming mice. In the second part of the study, involving SD rats, pathological alterations in the major organs (heart, liver, kidney and lungs) were observed in sepsis; however, following treatment with EPO the pathological alterations in the organs were significantly reduced, indicating that the use of EPO may improve the prognosis of sepsis and MODS, and therefore reduce mortality.

Hemodynamic indicators of the heart can comprehensively reflect the degree of heart damage following sepsis and the protective effect of drug intervention. Among these indicators, LVSP and +dP/dt_max_ are sensitive indicators of myocardial systolic function and −dP/dt_max_ is a sensitive indicator of myocardial diastolic function. In the present study it was demonstrated that the LVSP, +dP/dt_max_ and −dP/dt_max_ were significantly reduced in septic SD rats compared with those in sham-operated rats (P<0.01). In the present study, the observation of cardiac hemodynamics suggested that +dP/dt_max,_ −dP/dt_max_ and LVSP of the left ventricle in the septic rats was significantly reduced compared with that of the normal control group. The significant decrease of LVSP, +dp/dt max and −dp/dt max index of the CLP group appeared at 3 h and reached the lowest point at 6 h, which was significantly lower compared with that of the control group (P<0.01). The +dp/dtmax, −dp/dtmax and LVSP of the EPO rats was gradually restored. These results demonstrated that EPO assisted in the maintenance and recovery of cardiac systolic and diastolic function in rats with sepsis.

cTnI is an indicator that has been found to reflect the degree of myocardial injury after sepsis and the protective effect of drug intervention with high sensitivity and specificity (22,23). In the present study it was demonstrated that levels of cTnI were significantly increased in sepsis. The levels were highest at 12 h and then decreased; however, they remained significantly higher than those of the control group. The increase in cTnI levels indicates that there was myocardial damage when sepsis occurred; when the myocardial cells were damaged, the membrane permeability was increased and troponin moved out of the cells, thus elevating levels of troponin in the blood. The increase and then reduction in cTnI was due to the dynamic equilibrium between the release and degradation of troponin within the myocardial cell cytoplasm and the depletion of troponin (24). Therefore, it should not be assumed that, during sepsis, myocardial damage was reduced over time. Following treatment with EPO, the cTNI levels were significantly decreased and a significant promotive effect on hemodynamic parameters for left ventricular systolic and diastolic function were observed. This further indicates that EPO has a protective effect against myocardial injury in septic rats. In the clinic, one of the indicators for myocardial cell damage is change in myocardial enzymes. In the present study, alterations in serum CK were observed. Treatment with EPO significantly reduced the variation in serum CK values, suggesting that myocardial damage was reduced. The CK values increased at 3 h and decreased at 6 h after CLP, indicating that myocardial cell damage occurred in early sepsis, the compensatory ability of the body increased the heart function instead of decreasing it. CK increased again 12 h after surgery with a continuously increase trend, suggesting that the body was no longer in a compensatory stage of shock and the treatment of sepsis was more difficult. The results further suggested that, in accordance with the ‘Surviving Sepsis Campaign International Guidelines for Management of Severe Sepsis and Septic Shock, 2012’, treatment is required to be performed in early sepsis, including timely and reasonably conducted early goal-directed therapy (EGDT), which was particularly important in preventing the occurence of multiple organ failure in sepsis and reducing the mortality rate of sepsis.

The article "Protective effect of erythropoietin against myocardial injury in rats with sepsis and its underlying mechanisms" was retracted in 2025. Reasons: duplicated images; overlap with earlier publications; concerns about the images; concerns about the citations.

In the present study, pathological sections of the major organs (heart, liver, kidney and lungs) were observed. Under the light microscope, a large number of ruptured cardiac myofilaments, myocardial cell edema and severely damaged and disordered muscle fiber structures were observed in the heart 24 h after the CLP, as well as the infiltration of inflammatory cells into the myocardial tissue. Following treatment with EPO, the pathological damage to the heart was significantly reduced, and the degree of damage to the other major organs (liver, kidney and lungs) was also significantly reduced, suggesting that in the early treatment of sepsis, attention should be paid to the protection and support of the functions of the heart and other organs in order to prevent the occurrence of multiple organ failure and to reduce the sepsis-associated mortality rate.

CRP is an acute phase reactive protein expressed when acute inflammation occurs in the body; in the clinic, it is often used to monitor infectious diseases. The prognosis of sepsis and the inflammatory state of the body may be reflected by the level of serum CRP. In the present study, CRP was significantly increased 6 h after CLP, which further suggested that an inflammatory response occurred in the animal models. The levels of CRP decreased following treatment with EPO.

The results of this study demonstrated that, 3 h after the CLP, the levels of serum TNF-α and IL-6 in the CLP and EPO groups were significantly increased compared with those in the Sham group; however, the peak of the EPO group was lower compared with that of the CLP group. This suggests that excessive cytokine release occurred during the progression of sepsis and that a significant inflammatory response was present in the body during the early stages of sepsis. As an anti-inflammatory substance, EPO inhibits the release of TNF-α and IL-6 and therefore inhibits the excessive inflammatory response. As a result, EPO reduces the pathological damage caused by the inflammatory response of tissues and organs and acts to protect the myocardium. This is conducive to the prevention of the occurrence and development of MODS during sepsis, and therefore improves the prognosis of sepsis. In the present study, the serum levels of IL-10 were significantly increased at 3 h and reached a peak at 6 h, whilst the serum levels of TNF-α and IL-6 at 6 h were significantly reduced compared with those at 3 h after the CLP (P<0.05). After 12 h, the serum levels of IL-10 gradually decreased, and the serum levels of TNF-α and IL-6 also showed a declining trend, indicating that the inflammatory factors of septic rats were decreased by varying degrees. IL-10, as anti-inflammatory cytokine, inhibits the synthesis of proinflammatory cytokines, thus helping to reduce the systemic inflammatory response and restore the balance of the inflammatory response.

The results of this study demonstrated that, 24 h subsequent to sepsis injury, the early and late apoptosis rates of the heart, liver, kidney and lung cells in the EPO and CLP groups were significantly increased compared with those in the Sham group. The early apoptosis rate of the cells in the EPO group following injury was significantly lower than that of the cells in the CLP group. These results suggest that EPO may inhibit cardiomyocyte apoptosis following sepsis, and the administration of exogenous EPO may reduce cardiac apoptosis caused by septic damage.

The article "Protective effect of erythropoietin against myocardial injury in rats with sepsis and its underlying mechanisms" was retracted in 2025. Reasons: duplicated images; overlap with earlier publications; concerns about the images; concerns about the citations.

A potential mechanism underlying the inhibition of myocyte apoptosis by EPO is that EPO acts through the mitochondrial pathway. In the present study rhodamine 123 was used to detect alterations in mitochondrial membrane potential in the three groups using flow cytometric analysis. The results of the study confirmed that the mitochondrial function in the major organs was affected in sepsis, and that mitochondrial membrane potential was decreased. In the EPO group, the fluorescence peak was significantly shifted to the right in the rats cells of the major organs (heart, liver, kidney and lungs) and the fluorescence intensity of the cells was increased compared with the CLP group. This indicates that, in the EPO group, there was a significant attenuation in the reduction of mitochondrial membrane potential; thus, apoptosis was inhibited. These results suggest that EPO inhibits apoptosis through the mitochondrial pathway.

In the present study, the activation of NF-κB was examined by determining the expression levels of NF-κB p65 protein. The results demonstrated that the expression of NF-κB p65 protein in septic rats in the EPO and CLP groups was significantly increased compared with that in the rats in the Sham group. Following treatment with EPO, the expression of NF-κB p65 protein was significantly lower than that in the CLP group. The inflammatory pathology of the organs and tissues (heart, liver, kidney and lungs) in the septic rats was also significantly reduced. Combining the findings for the levels of TNF-α, IL-6 and IL-10, as well as the expression of CRP and NF-κB p65 protein, the results suggest that EPO decreased the expression of its downstream inflammatory mediators by inhibiting the activation of NF-κB, and, as a result, reduced the inflammatory damage to the heart tissue of septic rats. In addition, levels of the serum anti-inflammatory factor IL-10 were increased following intervention with EPO, which promoted the restoration of the anti-inflammatory balance; this was one of the mechanisms of inflammatory damage mitigation in the tissues of septic rats.

These anti-inflammatory and protective effects of EPO cells are consistent with previous studies in animal models of sepsis and inflammation. The pre-and post- use of EPO have been observed to inhibit injury. In an animal model of necrotizing pancreatitis, EPO reduces sepsis-induced acute lung injury and exhibits improved maintainence of microvascular cell integrity (1). In the treatment of patients with renal failure undergoing peritoneal dialysis (2), peripheral blood neutrophil count decreases, neutrophil activation is inhibited and inflammatory cytokines are reduced, demosntrating that EPO can inhibit the inflammatory response. It has also been suggested that inflammation in the central nervous system can be mitigated following application of EPO (3).

The article "Protective effect of erythropoietin against myocardial injury in rats with sepsis and its underlying mechanisms" was retracted in 2025. Reasons: duplicated images; overlap with earlier publications; concerns about the images; concerns about the citations.

In evaluating a new treatment program, the comparable side effects require consideration. The data of patients with renal failure indicated that, the risk of thrombotic events increased when hemoglobin exceeded 12g/L (25,26). The risk increased by 1.3% (27) in patients with acute myocardial infarction. This occurred when the hemoglobin concentration was <10g/L, indicating that the prothrombotic state was not entirely dependent on blood viscosity, but attributed to changes in platelets and endothelial cells (28). Microthrombosis can cause organ failure and sepsis coagulopathy (1,2) and EPO can worsen the situation. Disease in certain cancer patients can worsen as EPO increases the risk of thrombosis and may induce tumor progression (29), suggesting concern in the use of EPO following development of sepsis in malignant diseases. If EPO is used in the early stages of sepsis, undesirable side effects appear and more serious side effects, including poor development of red blood cells is caused by lack of EPOR in the body (28). Therefore, the side effects of using EPO clinically as a new method of treatment requires close observation.

In conclusion, sepsis is caused by the induction of the inflammatory cascade by endotoxin, resulting in the excessive release of inflammatory mediators from the body and leading to an imbalance of pro- and anti-inflammatory factors. This inflammatory response activates NF-κB. Therefore, treatment targeting only one or two types of inflammatory mediators is ineffective; in order to effectively inhibit the disease development and improve prognosis, intervention should be targeted against the transduction signals from the source. Therefore, NF-κB, the central factor of multiple inflammatory pathways, is an important target for treatment, and blocking the activation of NF-κB may prevent further deterioration caused by the disease. The results of this study showed that NF-κB is involved in the processes leading to the inflammation-induced tissue damage in septic rats. EPO inhibits NF-κB and regulates and promotes the anti-inflammatory balance, thereby alleviating tissue injury in septic rats and exhibiting a protective role. This provides a molecular mechanism of action for the application of EPO in the clinical treatment of sepsis. However, the potential side effects and inadequacies of EPO highlighted in the present study should be considered in the evaluation of a new treatment program. Data from patients with renal failure and acute myocardial infarction showed that the risk of thrombotic events was increased when the concentration of hemoglobin was >12 g/l (25,26). Furthermore, microthrombi can cause septic organ failure and coagulopathy, and EPO may aggravate this. The side effects should be closely observed in the use of EPO as a novel therapeutic treatment for sepsis.

The article "Protective effect of erythropoietin against myocardial injury in rats with sepsis and its underlying mechanisms" was retracted in 2025. Reasons: duplicated images; overlap with earlier publications; concerns about the images; concerns about the citations.

## Figures and Tables

**Figure 1:** Mortality of Kunming mice (%) over seven days after the surgery. Roc, Rocephin; CLP, cecal ligation and puncture; EPO, erythropoietin.

**Figure 2:** Dynamic changes in the myocardium (A) LVSP, (B) +dP/dt_max_ and (C) −dP/dt_max_ in the rats in each group. CLP, cecal ligation and puncture; EPO, erythropoietin; LVSP, left ventricular systolic pressure; +dP/dt_max_, rate of left ventricular pressure rise; −dP/dt_max_, rate of left ventricular pressure decline.

**Figure 3:** Dynamic changed in the serum (A) CRP, (B) TNF-α, (C) IL-6 and (D) IL-10 levels in the rats in each group. CLP, cecal ligation and puncture; EPO, erythropoietin; CRP, C-reactive protein; TNF-α, tumor necrosis factor α, IL, interleukin.

**Figure 4:** Dynamic changes in the serum levels of (A) cTnI, (B) CK, (C) AST and (D) LDH in the rats in each group. cTnI, cardiac troponin I; CK, creatine kinase; AST, aspartate aminotransferase; LDH, lactate dehydrogenase; CLP, cecal ligation and puncture; EPO, erythropoietin.

**Figure 5:** Comparison of the early apoptotic rates among the groups. Annexin V/fluorescein isothiocyanate was used to detect the early apoptosis rates of rat (Aa–d) cardiac myocytes and (Ba–d) liver, (Ca–d) kidney and (Da–d) lung cells of each group (Sham, EPO and CLP) 24 h after the CLP surgery. CLP, cecal ligation and puncture; EPO, erythropoietin.

**Figure 6:** Comparison of mitochondrial membrane potentials among the groups. Flow cytometric analysis was used to determine the mitochondrial membrane potential of rat (Aa–d) cardiac myocytes and (Ba–d) liver, (Ca–d) kidney and (Da–d) lung cells of each group (Sham, EPO and CLP) 24 h after the CLP surgery. CLP, cecal ligation and puncture; EPO, erythropoietin.

**Figure 7:** Comparison of NF-κB p65 expression levels among the groups. Flow cytometric analysis was used to determine the expression levels of NF-κB p65 in rat (Aa–d) myocardial, (Ba–d) liver, (Ca–d) kidney and (Da–d) lung tissues in each group (Sham, EPO and CLP) 24 h after the CLP surgery. CLP, cecal ligation and puncture; EPO, erythropoietin; NF-κB, nuclear factor κ-light-chain-enhancer of activated B cells.

**Figure 8:** Pathological sections of the (A) heart, (B) liver, (C) kidney and (D) lung from rats in each group (Sham, EPO and CLP) 24 h after the CLP surgery (hematoxylin and eosin staining; magnification, ×400). CLP, cecal ligation and puncture; EPO, erythropoietin.

The article "Protective effect of erythropoietin against myocardial injury in rats with sepsis and its underlying mechanisms" was retracted in 2025. Reasons: duplicated images; overlap with earlier publications; concerns about the images; concerns about the citations.

**Table I:** Mortality of Kunming mice over seven days after the surgery.

		Mortality rate (%)										
		
Group	n	12 h	24 h	36 h	48 h	60 h	72 h	84 h	96 h	5 days	6 days	7 days
Sham	35	0.00	0.00	0.00	0.00	0.00	0.00	0.00	0.00	0.00	0.00	0.00
Roc	35	0.00	11.43	11.43	17.14	17.14	28.57	28.57	28.57	28.57	28.57	28.57
CLP	35	40.00	57.14	68.57	80.00	100.00	100.00	100.00	100.00	100.00	100.00	100.00
EPO	35	25.71	40.00	45.71	68.57	82.86	88.57	91.43	94.29	97.14	100.00	100.00

Roc, Rocephin; CLP, cecal ligation and puncture; EPO, erythropoietin.

**Table II:** Cardiac hemodynamic indices of Sprague Dawley rats in each group at different time-points.

			Time (h)				
			
Group	n	Index	0	3	6	12	24
Sham	8	LVSP (mmHg)	187.5±5.8	176.3±4.5	189.5±3.6	184.3±9.5	169.7±4.6
		+dP/dt_max_ (mmHg/sec)	7632±117.3	6840±121.7	6021±103.6	6987±128.3	6957±149.6
		−dP/dt_max_ (mmHg/sec)	−6772±136.8	−5737±184.7	−5245±176.3	−5347±112.6	−5976±138.7
CLP	8	LVSP (mmHg)	180.1±7.2	102.1±5.3^a^	67.4±6.1^b^	85.6±8.9^c^	92.7±7.6^d^
		+dP/dt_max_ (mmHg/sec)	6953±134.7	4002±375.7^a^	2821±372.6^b^	4366±473.8^c^	4496±504.1^d^
		−dP/dt_max_ (mmHg/sec)	−4921±192.3	−3821±187.3^a^	−1351±151.3^b^	−3081±416.1^c^	−3321±490.1^d^
EPO	8	LVSP (mmHg)	179.6±8.7	132.2±5.0^e^	119.1±5.1^f^	135.4±6.7^g^	138.3±5.9^h^
		+dP/dt_max_ (mmHg/sec)	7055±101.9	5471±180.3^e^	5077±153.2^f^	5350±211.6^g^	5379±143.9^h^
		−dP/dt_max_ (mmHg/sec)	−5053±152.2	−4546±112.1^e^	−4121±149.5^f^	−4214±109.2^g^	−4350.3±173.1^h^

Results are presented as the mean ± standard deviation. Comparison among the CLP, EPO and Sham groups (^a^P<0.01, ^b^P<0.01, ^c^P<0.01 and ^d^P<0.01). Comparison between the EPO and the CLP groups (^e^P<0.01, ^f^P<0.01, ^g^P<0.01 and ^h^P<0.01). CLP, cecal ligation and puncture; EPO, erythropoietin; LVSP, left ventricular systolic pressure; +dP/dt_max_, rate of left ventricular pressure rise; −dP/dt_max_, rate of left ventricular pressure decline.

**Table III:** Inflammatory reaction indices of Sprague Dawley rats in each group at different time-points.

			Time (h)				
			
Group	n	Index	0	3	6	12	24
Sham	8	CRP (mg/l)	0.91±0.15	1.01±0.18	1.00±0.16	1.05±0.14	1.00±0.09
		TNF-α (ng/l)	11.68±0.87	12.92±0.91	13.65±5.02	12.87±4.36	11.96±4.75
		IL-6 (ng/l)	67.23±24.36	68.71±11.48	70.21±50.32	74.33±23.14	66.98±45.12
		IL-10 (pg/ml)	47.65±11.32	49.91±10.34	51.21±11.45	53.64±23.87	61.25±34.69
CLP	8	CRP (mg/l)	0.98±0.09	1.26±0.18	2.31±0.33^b^	1.89±0.29^c^	1.41±0.26
		TNF-α (ng/l)	13.32±0.22	63.69±6.85^a^	45.58±3.96^b^	41.46±5.04^c^	25.99±5.08^d^
		IL-6 (ng/l)	70.46±41.26	1768.93±195.11^a^	958.71±141.59^b^	449.91±56.28^c^	198.05±58.02^d^
		IL-10 (pg/ml)	48.99±14.01	198.62±42.12^a^	711.26±84.97^b^	528.65±108.71^c^	334.17±44.17
EPO	8	CRP (mg/l)	0.89±0.11	1.12±0.13	1.86±0.23^f^	1.45±0.21^g^	1.17±0.15
		TNF-α (ng/l)	12.53±0.36	53.57±5.48^e^	33.31±4.21^f^	29.44±2.68^g^	17.98±2.13^h^
		IL-6 (ng/l)	66.96±30.12	1129.49±151.26^e^	666.53±191.46^f^	309.32±65.44^g^	122.41±34.54^h^
		IL-10 (pg/ml)	50.81±13.65	297.82±43.17^e^	1345.64±171.51^f^	798.78±61.36^g^	392.25±52.79

Results are presented as the mean ± standard deviation. Comparison among the CLP, EPO and Sham groups (^a^P<0.01, ^b^P<0.01, ^c^P<0.01 and ^d^P<0.01). Comparison between the EPO and the CLP groups (^e^P<0.01, ^f^P<0.01, ^g^P<0.01 and ^h^P<0.01). CLP, cecal ligation and puncture; EPO, erythropoietin; CRP, C-reactive protein; TNF-α, tumor necrosis factor α, IL, interleukin.

The article "Protective effect of erythropoietin against myocardial injury in rats with sepsis and its underlying mechanisms" was retracted in 2025. Reasons: duplicated images; overlap with earlier publications; concerns about the images; concerns about the citations.

**Table IV:** Serum myocardial enzymology indices of Sprague Dawley rats in each group at different time-points.

			Time (h)				
			
Group	n	Index	0	3	6	12	24
Sham	8	cTnI (ng/ml)	0.009±0.004	0.013±0.009	0.021±0.017	0.012±0.004	0.036±0.018
		CK (U/l)	436.12±97.38	732.25±107.48	689.47±98.56	807.24±78.14	825.48±87.63
		AST (U/l)	225.68±68.33	264.27±95.27	278.29±87.96	299.18±75.64	324.29±89.67
		LDH (U/l)	725.15±87.63	762.66±96.17	788.57±101.32	800.68±99.68	795.51±55.36
CLP	8	cTnI (ng/ml)	0.024±0.012	0.386±0.171	1.184±0.385^b^	2.321±0.447^d^	1.173±0.249^e^
		CK (U/l)	457.31±88.48	4632.51±638.39^a^	2704.75±415.82^c^	8638.75±1995.43^d^	10604.12±3660.05^e^
		AST (U/l)	246.35±78.36	582.55±213.54	1233.87±429.12^c^	1865.24±349.14^d^	2543.36±598.43
		LDH (U/l)	802.65±79.54	1282.12±357.66	1755.25±446.28	2945.87±744.92^d^	4246.51±771.87
EPO	8	cTnI (ng/ml)	0.018±0.009	0.344±0.113	0.672±0.349^g^	1.134±0.247^i^	0.878±0.184^k^
		CK (U/l)	482.42±68.36	2580.25±941.62^f^	1638.36±750.83^h^	6060.63±1766.55^j^	8728.75±1975.09^k^
		AST (U/l)	267.26±88.94	546.75±127.86	743.52±107.22^h^	1199.12±217.06^i^	2445.37±774.83
		LDH (U/l)	767.34±95.66	1035.51±189.45	1319.12±527.93	1933.12±546.25^i^	4073.37±552.56

Results are presented as the mean ± standard deviation. Comparison among the CLP, EPO and Sham groups (^a^P<0.01, ^b^P<0.01, ^c^P<0.01, ^d^P<0.01 and ^e^P<0.01). Comparison between the EPO and CLP groups (^f^P<0.01, ^g^P<0.05, ^h^P<0.01, ^i^P<0.01, ^j^P<0.05 and ^k^P<0.05). CLP, cecal ligation and puncture; EPO, erythropoietin; cTnI, cardiac troponin I; CK, creatine kinase; AST, aspartate aminotransferase; LDH, lactate dehydrogenase.
